This article has been retracted.

# Investigation on Health Promotion by the Typical Sports for Teenagers with Self-Efficacy and Sports Commitment Questionnaires

**DOI:** 10.1155/2021/8677182

**Published:** 2021-08-31

**Authors:** Qiaoyin Tan, Weide Shao

**Affiliations:** ^1^College of Teacher Education, Zhejiang Normal University, Jinhua, Zhejiang 321004, China; ^2^College of Physical Education and Health Sciences, Zhejiang Normal University, Jinhua, Zhejiang 321004, China

## Abstract

This work studied the health promotion by the typical sports using self-efficacy and sports commitment questionnaires for 804 teenagers, who were from different interest-oriented sport classes. Five typical interest-oriented sport classes were selected due to the difference in sport characteristics: basketball, swimming, tennis, taekwondo, and archery. Statistical analyses, ANOVA analysis, and multiple comparisons (with least significant difference, LSD) were applied to the collected data. It has been found that boys and girls have similar self-efficacy of adolescent sports health. Adolescents' self-efficacy of sports health has significant differences among different sports items, where the basketball group scored the highest. Adolescents in the professional level have the highest self-efficacy of sports health, whereas the skillful level and beginner level have no significant difference. The male students are more enthusiastic and fond of sports than female students. There are significant differences between sports commitment and sports health of adolescents in different sports, where the basketball group scored the highest. Exercise induces higher score of sports commitment; however, no significant difference is observed for the skillful level and the beginner level. The significant positive correlation is found between sports health and self-efficacy and sports commitment, self-efficacy, and sports commitment. Besides, the role of self-efficacy is partial intermediary between sports health and sports commitment.

## 1. Introduction

Choosing an active lifestyle is the priority trend of health. A large number of studies have shown that, besides the prevention of diseases and the treatment after discovery [1], physical exercise is an effective means to promote health [2, 3]. Adult-based research shows that there is a developmental positive correlation between sports level and physical health [4–6]. Among teenagers, periodic sports also have a positive impact on health [7]. Improving the level of physical activity is one of the main intervention strategies to improve adolescent health [8].

There are several longitudinal studies on the health promotion of teenagers in sports clubs. These studies show that promoting the positive development of teenagers through sports is the future direction of health promotion [9]. Sports clubs are an ideal environment for children and adolescents to promote health [10]. Some studies have found that the establishment of healthy sports clubs is a conceptual mapping method to effectively improve the quality of life [11]. Some government-led health and welfare programs promote the health of club members significantly [12].

As far as we know, China has not studied the relationship between various typical sports and health status of teenagers, and the current research aims to fill this gap. Based on the sport characteristics, we choose five typical sports as the studying objects, including basketball, swimming, tennis, taekwondo, and archery. Skill-oriented sports include basketball in the same field [13], tennis across the net [14], taekwondo in fighting [15], and archery in performance accuracy [16]. Swimming is chosen by the class dominated by physical ability [17]. The purpose of this study is to evaluate the relationship between typical exercise and health promotion. To investigate teenagers' sports-related behaviors in clubs, the work is carried out to find out the details of their self-efficacy and action feelings and to analyze their promotion effect on health behaviors. Math tools have been widely used in the analysis of healthcare data, including statistical analysis [18–21], computer techniques (i.e., molecular docking) [22, 23], and artificial intelligence [24]. In this work, math tools have been used for the comprehensive healthcare analysis.

## 2. Methods

### 2.1. Object

Table 1 shows the basic statistics of the investigation. 804 teenagers from different interest-oriented sport classes were online investigated using the questionnaire (in the supplementary file). Five typical interest-oriented sport classes were selected due to the difference in sport characteristics: basketball, swimming, tennis, taekwondo, and archery. The levels of professional, skillful, and beginner are determined according to the questionnaire results with subjective answers. Self-efficacy and sports commitment questionnaires [25] were filled by the object. ANOVA analysis [26] was applied to the collected data.

## 3. Results and Discussion

### 3.1. Analysis on the Current Situation of Self-Efficacy in Sports Health

Table 2 shows the comparison of the difference of self-efficacy in sports health between different genders (independent sample t-test).  Table 3 shows the self-efficacy analysis for different genders. The results of the independent sample t-test on the self-efficacy of sports health of teenagers of different genders showed that the statistical quantity *t* = −0.313 and the significance level *P* = 0.632 > 0.05, indicating that there is no significant difference between boys and girls in the self-efficacy of adolescent sports health; that is, both boys and girls have similar self-efficacy. In addition, it can be seen from the description table that there are 464 boys among 804 teenagers participating in the questionnaire. 340 female students and their self-efficacy scores averaged 3.95 and 3.98, respectively, which were basically the same.

Table 4 shows the comparison of Self-efficacy of adolescents in different sports (one-way ANOVA analysis).  Table 5 shows the self-efficacy analysis for different sports. One-way ANOVA results for self-efficacy of sports health of adolescents in different sports items showed that statistical *F* = 3.321 and significance level *P* = 0.010 < 0.05, indicating that, at the significance level of 5%, adolescents' self-efficacy of sports health has significant differences among different sports items. It can be seen from the description table that, among the 804 teenagers who participated in the questionnaire, 253 are from taekwondo, and the average self-efficacy score of this project is 3.96. The least is swimming teenagers, with 119 teenagers, and the average score is 3.89. Among them, basketball sport has the highest average score, with the average score of 4.14.

Table 6 shows the multiple comparisons (with least significant difference, LSD) to see the differences between the various sports. The results in the table show that the *P* values of significance between basketball and swimming, tennis, taekwondo, and archery are 0.003, 0.001, 0.012, and 0.017, respectively, all less than 0.05, indicating that there are significant differences in the sense of self-efficacy of the youth's sports health between basketball and swimming, basketball and tennis, basketball and taekwondo, and basketball and archery.

Table 7 shows the comparison of self-efficacy of adolescents with different sports levels in sports health with ANOVA.  Table 8 shows the self-efficacy analysis for different exercise levels. One-way ANOVA was carried out on the self-efficacy of sports health of adolescents at different sports levels. The results showed that the statistical quantity *F* = 31.045, and the significance level *P* < 0.05, indicating that the self-efficacy of sports health of adolescents at the significance level of 5% was significantly different among different sports levels. It also can be seen from the description table that, among the 804 teenagers who participated in the questionnaire, 436 of them are in the stage of beginners, with an average of 3.89, 143 of them are in the professional level, and 225 of them are in the skillful level, with an average of 4.36 and 3.85, respectively. From the mean value, it can be seen that adolescents in the professional level have the highest self-efficacy of sports health. Subsequently, we used multiple comparisons (with least significant difference, LSD) to look at the differences between the exercise levels.

Table 9 shows the multiple comparisons (LSD) for differences in exercise levels. The results of multiple comparisons showed that the significance level *P* values between the professional level and the skillful level, the professional level, and the beginner level are all ≤0.001, which is less than 0.05, indicating that there are significant differences in self-efficacy between the professional level and the skillful level and between the professional level and the beginner level. The significance level between the skillful level and the beginner level is *P* = 0.408 > 0.05. The results showed that there was no significant difference between the skillful level and the beginner level in the self-efficacy of adolescents' sports health.

### 3.2. Analysis on the Current Situation of Exercise Commitment of Adolescent Sports Health

Table 10 shows the comparison of the differences of exercise commitment in sports health among adolescents of different genders (independent sample t-test).  Table 11 shows the sports commitment for different genders. The results of the independent sample t-test on exercise health and exercise commitment of adolescents of different genders showed that the statistical quantity *t* = 1.959 and the significance level *P* = 0.044 < 0.05, indicating that, at the significance level of 5%, there is a significant difference between boys' and girls' sports commitment in adolescent sports health. In addition, it can be seen from the description table that the mean value of 464 boys' sports commitment among 804 teenagers participating in the questionnaire is 4.11. The average of 340 female students' sports commitment was 4.01, and the score of male students' sports commitment was significantly higher than that of female students, indicating that male students are more enthusiastic and fond of sports than female students.

Table 12 shows the comparison of differences in exercise commitment of adolescents in different sports using ANOVA.  Table 13 shows the sports commitment for different sport types. One-way ANOVA analysis of sports commitment for sports health of adolescents in different sports shows that *F* = 2.812 and significance level *P* = 0.025 < 0.05, indicating that there are significant differences between sports commitment and sports health of adolescents in different sports at the significance level of 5%. From the description table, it can be seen that, among the 804 teenagers who participated in the questionnaire, the highest mean value is that of 151 teenagers who participated in basketball sports, reaching 4.21, followed by swimming and taekwondo, both of which are 4.06, and the lowest is that of archery, only 3.99. Subsequently, we used multiple comparisons (LSD) to look at the differences of exercise commitment among different sports.

Table 14 shows the multiple comparisons (LSD) for differences in sports commitment among different sports. Multiple comparison results showed that the *P* values of significance level between basketball and tennis, taekwondo, and archery were 0.013, 0.034, and 0.011, respectively, which were all less than 0.05, indicating that, at the significance level of 5%, there were significant differences in the self-efficacy of adolescent sports health between basketball and tennis, basketball and taekwondo, and basketball and archery. There was no significant difference between basketball and swimming, *P* = 0.076 > 0.05.

Table 15 shows the comparison of differences in sports commitment among adolescents with different sports levels in sports health using ANOVA.  Table 16 shows the sports commitment for different sports levels. One-way ANOVA was conducted for sports commitment of adolescents with different sports levels. The results showed that *F* = 21.747 and significance level *P* < 0.05, indicating that, at the significance level of 5%, there was a significant difference in sports commitment of adolescents with different sports levels. It also can be seen from the description table that, among the 804 teenagers who participated in the questionnaire, 436 of them are in the stage of beginner, with an average value of 3.97. The average value of sports commitment of 143 teenagers in the professional level is the highest, reaching 4.42. The average value of the last 225 teenagers in the skillful level is 4.02. From the mean value, it can be seen that the sports health commitment of adolescents in the professional level is the highest, followed by skillful level, and the lowest among those beginners. This indicates that exercise induces higher score of sports commitment. Subsequently, we used multiple comparisons (LSD) to look at the differences between the sports levels.

Table 17 shows the multiple comparisons (LSD) for different the sports levels. The results of the abovementioned multiple comparisons show that the significance *P* values between professional and skillful and between professional and beginner level are all ≤0.001, which is less than 0.05, indicating that there are significant differences between professional and skillful and between professional and beginner. The significance level between skillful and beginner level is *P* = 0.494 > 0.05. The results showed that there was no significant difference between the skillful and the beginner level of sports commitment in the adolescents' sports health.

### 3.3. Correlation and Regression-Mediation Analysis

Table 18 shows the correlation analysis for sports health, self-efficacy, and sports. Correlation analysis [27] is performed in the questionnaire work for sports health, self-efficacy, and sports commitment. The correlation analysis of sports health and self-efficacy and sports commitment shows a significant correlation between youth sports health and sports commitment, significant activity level *P* < 0.05, and Pearson correlation coefficients are 0.856, 0.815, and 0.662, respectively, indicating a significant positive correlation between sports health and self-efficacy and sports commitment, self-efficacy, and sports commitment.

Table 19 shows the regression-mediation analysis for sports health, self-efficacy, and sports commitment. Regression-mediation analysis [28] is performed in the questionnaire work for sports health, self-efficacy, and sports commitment. From the abovementioned analysis results, the significance level of *P* ≤ 0.001 < 0.05 is passed between sports health and sports commitment. The regression coefficient is of 0.206. The regression coefficient between sports health and sports commitment is 0.189, less than the regression coefficient of model 1, indicating the role of self-efficacy is partial intermediary between sports health and sports commitment.

## 4. Conclusions

In this work, investigation and analysis were carried out on the health promotion by the typical sports using self-efficacy and sports commitment questionnaires for 804 teenagers, who were from different interest-oriented sport classes. Five typical interest-oriented sport classes were selected due to the difference in sport characteristics: basketball, swimming, tennis, taekwondo, and archery. Statistical analysis, ANOVA analysis, and multiple comparisons (LSD) were applied to the collected data. Some findings from the analysis include (1) boys and girls have similar self-efficacy of adolescent sports health; (2) adolescents' self-efficacy of sports health has significant differences among different sports items, where the basketball group scored the highest; (3) adolescents in the professional level have the highest self-efficacy of sports health, whereas the skillful level and beginner level have no significant difference; (4) male students are more enthusiastic and fond of sports than female students; (5) there are significant differences between sports commitment and sports health of adolescents in different sports, where the basketball group scored the highest; (6) exercise induces higher score of sports commitment; however, no significant difference is observed for the skillful level and the beginner level; (7) significant positive correlation between sports health and self-efficacy and sports commitment, self-efficacy, and sports commitment; and (8) the role of self-efficacy plays a partial intermediary between sports health and sports commitment.

## Figures and Tables

**Table 1:** Basic statistics of the investigation.

Name	Classification	Frequency	Percentage (%)
Gender	Male	464	57.7
	Female	340	42.3

Sports	Basketball	151	18.8
	Swimming	119	14.8
	Tennis	148	18.4
	Taekwondo	253	31.5
	Archery	133	16.5

Sports grade	Professional	143	17.8
	Skillful	225	28
	Beginner	436	54.2

**Table 2:** Comparison of the difference of self-efficacy in sports health between different genders (independent sample t-test).

		Levene's test for the equation of variance		The t-test for the mean value equation						
		F	Sig.	t	df	Sig. (bilateral)	MD	SD	95% confidence interval	
									Lower	Upper
Self-efficacy	Assuming the variance is equal	19.583	0.000	−0.465	802	0.642	−0.02311	0.04973	−0.12074	0.07451
	Assuming the variance is not equal			−0.478	790.356	0.632	−0.02311	0.04831	−0.11795	0.07172

**Table 3:** Self-efficacy analysis for different genders.

Self-efficacy	*N*	M±SD	t	*P*
Male	464	3.95 ± 0.75	−0.478	0.632
Female	340	3.98 ± 0.34		

**Table 4:** Comparison of self-efficacy of adolescents in different sports (one-way ANOVA analysis).

	Quadratic sum	df	Mean square	F	Sig.
Interblock	6.368	4	1.592	3.321	0.010
Within the group	382.981	799	0.479		
Total	389.349	803			

**Table 5:** Self-efficacy analysis for different sports.

Self-efficacy	*N*	M±SD	F	*P*
Basketball	151	4.14 ± 0.69	3.321	≤0.001
Swimming	119	3.89 ± 0.64		
Tennis	148	3.88 ± 0.70		
Taekwondo	253	3.96 ± 0.74		
Archery	133	3.94 ± 0.70		

**Table 6:** Multiple comparisons (with least significant difference, LSD) to see the differences between the various sports.

(I) sports	(J) sports	MD (I-J)	SE	*P*
Basketball	Swimming	0.24903^*∗*^	0.08487	0.003
	Tennis	0.25805^*∗*^	0.08008	≤0.001
	Taekwondo	0.17938^*∗*^	0.07120	0.012
	Archery	0.19758^*∗*^	0.08233	0.017

**Table 7:** Comparison of self-efficacy of adolescents with different sports levels in sports health with ANOVA.

	Quadratic sum	df	Mean square	F	Sig.
Interblock	28.009	2	14.005	31.045	0.000
Within the group	361.340	801	0.451		
Total	389.349	803			

**Table 8:** Self-efficacy analysis for different exercise levels.

Self-efficacy	N	M±SD	F	*P*
Professional	143	4.36 ± 0.62	31.045	≤0.001
Skillful	225	3.85 ± 0.72		
Beginner	436	3.89 ± 0.70		

**Table 9:** Multiple comparisons (LSD) for differences in exercise levels.

(I) sports grade	(J) sports grade	MD (I-J)	SD	*P*
Professional	Skillful	0.51549^*∗*^	0.07183	≤0.001
	Beginner	0.46988^*∗*^	0.06472	≤0.001

Skillful	Professional	−0.51549^*∗*^	0.07183	≤0.001
	Beginner	−0.04561	0.05513	0.408

Beginner	Professional	−0.46988^*∗*^	0.06472	≤0.001
	Skillful	0.04561	0.05513	0.408

**Table 10:** Comparison of the differences of exercise commitment in sports health among adolescents of different genders (independent sample t-test).

		Levene's test for the equation of variance			The t-test for the mean value equation					
		F	Sig.	t	df	Sig. (bilateral)	MD	SD	95% confidence interval	
									Lower	Upper
Sports commitment	Assuming the variance is equal	14.359	0.000	1.915	802	0.056	0.09916	0.05177	−0.00246	0.20078
	Assuming the variance is not equal			1.959	780.647	0.044	0.09916	0.05062	−0.00021	0.19852

**Table 11:** Sports commitment for different genders.

Sports commitment	*N*	M ± SD	t	*P*
Male	464	4.11 ± 0.77	1.959	0.044
Female	340	4.01 ± 0.66		

**Table 12:** Comparison of differences in exercise commitment of adolescents in different sports using ANOVA.

	Quadratic sum	df	Mean square	F	Sig.
Interblock	7.154	4	1.789	2.812	0.025
Within the group	508.144	799	0.636		
Total	515.298	803			

**Table 13:** Sports commitment for different sport types.

Sports commitment	N	M ± SD	F	*P*
Basketball	151	4.21 ± 0.71	2.812	0.025
Swimming	119	4.06 ± 0.63		
Tennis	148	4.01 ± 0.72		
Taekwondo	253	4.06 ± 0.75		
Archery	133	3.99 ± 0.78		

**Table 14:** Multiple comparisons (LSD) for differences in sports commitment among different sports.

(I) sports	(J) sports	MD (I-J)	SD	*P*
Basketball	Swimming	0.15799	0.08878	0.076
	Tennis	0.20826^*∗*^	0.08378	0.013
	Taekwondo	0.15792^*∗*^	0.07448	0.034
	Archery	0.21958^*∗*^	0.08613	0.011

**Table 15:** Comparison of differences in sports commitment among adolescents with different sports levels in sports health using ANOVA.

	Quadratic sum	df	Mean square	F	Sig.
Interblock	21.821	2	10.911	21.747	0.000
Within the group	401.876	801	0.502		
Total	423.698	803			

**Table 16:** Sports commitment for different sports levels.

Sports commitment	*N*	M ± SD	F	*P*
Professional	143	4.42 ± 0.63	21.747	≤0.001
Skillful	225	4.02 ± 0.73		
Beginner	436	3.98 ± 0.72		

**Table 17:** Multiple comparisons (LSD) for different sports levels.

(I) sports grade	(J) sports grade	MD (I-J)	SD	*P*
Professional	Skillful	0.40223^*∗*^	0.07575	≤0.001
	Beginner	0.44205^*∗*^	0.06826	≤0.001

Skillful	Professional	−0.40223^*∗*^	0.07575	≤0.001
	Beginner	0.03982	0.05814	0.494

Beginner	Professional	−0.44205^*∗*^	0.06826	≤0.001
	Skillful	−0.03982	0.05814	0.494

**Table 18:** Correlation analysis for sports health, self-efficacy, and sports commitment.

		Sports health	Self-efficacy	Sports commitment
Sports health	Pearson correlation	1	0.856^*∗∗*^	0.815^*∗∗*^
	Significance (bilateral)		0.000	0.000
	*N*	804	804	804

Self-efficacy	Pearson correlation	0.856^*∗∗*^	1	0.662^*∗∗*^
	Significance (bilateral)	0.000		0.000
	*N*	804	804	804

Sports commitment	Pearson correlation	0.815^*∗∗*^	0.662^*∗∗*^	1
	Significance (bilateral)	0.000	0.000	
	*N*	804	804	804

^*∗∗*^Significant correlation at 0.01 levels (bilateral).

**Table 19:** Regression-mediation analysis for sports health, self-efficacy, and sports commitment.

Model		Nonstandardized factor		Standard factor	t	Sig.
		B	Standard error	Trial version		
1	(Constant)	14.785	0.883		16.750	0.000
	Sports commitment	8.189	0.206	0.815	39.809	0.000

2	(Constant)	8.735	0.639		13.673	0.000
	Sports commitment	4.444	0.189	0.442	23.575	0.000
	Self-efficacy	5.557	0.185	0.563	29.997	0.000
Model 1: *R* = 0.815, *R*_2_ = 0.664, adjustment *R*_2_ = 0.664, *F* = 1584.754, *P* ≤ 0.001						
Model 2: *R* = 0.917, *R*_2_ = 0.842, adjustment *R*_2_ = 0.841, *F* = 2130.313, *P* ≤ 0.001						

^a^Dependent variable: sports health.

## Data Availability

All data used to support the findings of this study are included within the article and the supplementary file.

## Supplementary Materials

Supplementary Materials The questionnaire method and the collected raw questionnaire data for analysis are shown in the supplementary files.
